# Controlled Light Cross-Linking Technique to Prepare Healable Materials

**DOI:** 10.3390/polym9060241

**Published:** 2017-06-21

**Authors:** Soliman Abdalla, Fahad Al-Marzouki, Abdullah Obaid, Fatma Bahabri

**Affiliations:** Department of Physics, Faculty of Science, King Abdulaziz University Jeddah, P.O. Box 80203, Jeddah 21589, Saudi Arabia; fmphy@kau.edu.sa (F.A.-M.); soulimanabd@hotmail.com (A.O.); fbahabri@kau.edu.sa (F.B.)

**Keywords:** light, furan, healable materials, maleimide, poly(lauryl methacrylate)

## Abstract

Detection of defects, damages and cracks in structural polymers is very difficult, and even if they are detected, they will be very hard to be repaired. This is because different kinds of stress can reduce the mechanical efficiency of structural and functional thermosetting composite materials and they can damage the polymer matrix, thus reducing the purposed properties. General healing processes use thermal energy “alone” to heal these materials, thus impairing the intended properties of the materials. Therefore, we present a thermal healing ability that can be switched-on and/or -off at desire using illumination by photon energy (visible and ultra violet). By this technique, one can control local heal while keeping the efficiency of the material nearly unchanged. Furan-based cross-linker chemically reacts (forward- and reverse-reaction) with short-chains of maleimide-substituted poly(lauryl methacrylate) to form robust chemical bonds. This permits us to perform local control over thermally induced de- and/or re-cross-linking techniques. One can extend and apply this technique to cover micro-devices, coating-techniques, fine lithography, micro- and nano-fabrication processes, etc. Therefore, the present work developed a suitable technology with structural polymeric material, which has the ability to self-heal cracks (and damages) and recover structural function.

## 1. Introduction

Structural polymers are sensitive to damage, which results in mechanical degradation of fiber-reinforced polymer composites. This important problem leads to electrical failure in microelectronic-polymeric components. In particular, thermal energy and mechanical stresses could result in permanent and long-term problems in structural polymers and adhesive ones. In addition, the recent accelerated technologies are seeking for more efficient materials, which have the ability to self-repair inflicted damage. Moreover, several authors have studied cross-linking processes in order to get useful highly cross-linked polymers (CLPs), which used as matrices for structural adhesives [1], foamed structures composites [2], insulators for electronic packaging [3], etc. One can get excellent mechanical properties from these CLPs, for example high modulus, high fracture strength, and solvent resistance. However, the formation and propagation of cracks can permanently damage these materials by high stresses [4,5]. Recently, the exploration of self- healing of polymeric materials (and re-mending them) has become important subject in order to get self-healing material [6,7,8,9]. Polymeric chain entanglements occur with different intermolecular noncovalent interactions cause mending. Wang et al. and others have reported that small molecules can ensure crack healing in some thermoplastics [10,11]. In addition, Structural polymers are very sensitive to any deterioration such as cracks or structural-defects that are present through initial preparing technique. By using supramolecular polymers, or some dynamic covalent chemistry, one can introduce reversible connections in the polymer structure. In particular, the reversible Diels–Alder chemical reaction of furans with maleimides is widely known [12,13]. This reaction needs no more catalysts and it results in useful secondary products, which leads to enhancing the cross-linking mechanisms at simple conditions such as ambient conditions. At high temperatures, thermal reordering processes can restore the possible defect made during preparation. Thermal energy repairs and, therefore, healing processes happens under the conditions that some domains through the material either are difficult to repair or are destroyed [14]. Different physical and/or chemical processes such as mechanical stress [15], physical stimuli [16], pH variations [17,18] or redox changes [19] are useful in activation of polymers healing or repairing ability. We propose using light at ambient conditions in order to provide molecules with sufficient energy and locally control thermal healing processes. In order to overcome the difficulty of continuous need of light power, we propose applying a set of photons switchable reactants [20]. These switchable reactants are group of photons with sufficient energy to perform reversible cross-linking reaction (RCLR) (X_ON_ + P → X#P_ON_). This includes connecting and disconnecting polymer chains (P) by light photons energy.

When we complete healing processes with continuous light or UV irradiation, we noticed that if the dynamic covalent reaction is inhibited, CLP–X#P_ON_ and free cross-linker X_ON_ will be transform to their corresponding locked states (X_OFF_ and X#P_OFF_). This means that we can select to re-activate the polymer dynamic feature, which will result in reversibly switchable dynamic covalent developed composite.

We constructed our set ups on photo-switchable actions, which depend on reversible Diels–Alder reactions with maleimide. In particular, we used the heterocyclic organic furan, which contains diarylethene photo-switches. These compounds assure good bi-stability of the switchable material, thus we can deal with healing processes independently and selectively using visible light and ultraviolet.

## 2. Materials and Methods

### 2.1. General Procedure for Preparation of Cross Linkers (X#P_ON_ and X#P_OFF_)

1. In argon ambient: We dissolved co-polymer P (1.0 equivalent maleimide side-chains) and cross-linker X_ON_ (0.7 equivalent furan termini) in a minimum amount of dry tetra-hydro-furan (THF) in a 2.5 mL vial.
2. Then, we drop-casted onto a glass slide (GS) positioned in a Schlenk flask.
3. We pursuit this by immediate evacuation of Schlenk flask.
4. In order to get rid of residual solvent and to anneal the polymer mixture, we heated the evacuated-Schlenk flask (ESF) at 130 °C for 1.5 h.
5. In ESF, at room temperature, we carried out thermal cross-linking for about 16 h.
6. Then, we perform drop casting on to steel plates, for rheology.
7. We irradiate about 50% of the material using a LED XSL-365 nm-5E (Roithner Laser TecchnikGmbH, Vienna, Austria,) with electric polarization 4.2 V for LED under electric current 20 mA. The distance is about 3 cm normal to the sample. We kept the locked polymer network sample X#P_OFF_ for more analysis.
8. For about 2 h, we used LED Engin-460 nm-Blue Emitter LZ4/00B208 (Roithner Laser TecchnikGmbH, Vienna, Austria) with electric polarization 12 V for LED under electric current 2–3 mA to irradiate the locked and heated polymer films. The relatively long period of time (2 h) allows more examining of the reestablishment of the healability.

### 2.2. Scratching Techniques for Blocking Cross-Linker and Un-Blocking Cross-Linker (X#P_ON_ and X#P_OFF_)

We carried out scratches in the mm-range using a scalpel in a controlled manner. Then, we mask about 50% of the scratch and CLPs film X#P_ON_ using Al thin foil. In argon ambient, we illuminated the unmasked area in a Schlenk flask for 30 min. Then, we carried out suitable adjustment using the above-mentioned Roithner 365 nm in a distance of 3 cm normal to the GS to prepare X#P_OFF_. Then we removed the Al thin foil and heated the GS gradually from 27 up to 124 °C on a Deben Enhanced Cool stage in a sample chamber vacuum (B30–50 Pa) of a SEM TM-1000 control unit remaining at that temperature for 5 min For 2 h, we irradiated the material using LED 460 nm Engin-Emitter. Under similar conditions as for locking the polymer, we heated again for 2 h. After carrying out each step, we carried out FT-IR spectra and optical micrographs.

For work under inert conditions, HPLC grade solvents (Acros, Sigma-Aldrich, Gillingham Dorset, UK) were dried and degassed via a Pure Solv solvent purification system from Innovative Technologies (Gillingham Dorset, UK). Dried and degassed glassware was flushed with argon several times. Work with diarylethene-type compounds was done under red light. Liquid-NMR spectra were obtained on a 500 MHz (126 MHz for ^13^C) Bruker AVANCE II 500 spectrometer (Billerica, MA, USA) or on a 300 MHz (75 MHz for ^13^C) Bruker DPX 300 spectrometer (Billerica, MA, USA) at 25 °C.

### 2.3. Optical Micrographs

They were either acquired on a Bruker A670 Hyperion FT-IR microscope (Billerica, MA, USA) in the reflection mode with a visible objective, 40-times magnified (10× ocular, 4× vis-objective, for micrographs in main article) or with the optical detection unit of the atomic force microscope (AFM) facility (for micrographs presented in Figure 1a,b). The white balance of all images was automatically adjusted with a macro written for the Fiji software, provided by the light microscopy facility of the Cambridge Institute for Cancer Research, Cambridge, UK.

### 2.4. Fourier-Transform Infrared (FTIR) Spectroscopy

FT-IR was carried out on a Bruker Vertex (Billerica, MA, USA) 70v equipped with a Specac Golden Gate single reflection diamond ATR sample holder. Scans (number of scans: 128) were collected with a resolution of 4 cm^−1^ from 4000 to 400 cm^−1^. Baseline correction was performed using spline interpolation in (OLCN-USA).

### 2.5. Synthesis of Cross-Linker X_ON_

Using digital asset exchange software (DAE, Alpha point, San Francisco, CA, USA), the tetrafuryl-substituted DAE-type cross-linker X_ON_ was synthesized via a Suzuki cross coupling reaction of the precursor DAE15 with I where I is illustrated in Scheme 1. 

A five-step synthesis including a Michael-type addition yields the precursor DAE (1(3(2,5-dimethylfuryl))-2-(3-(5-chloro-2-methylthienyl)-cyclopentene, whose synthesis was recently described by our research group [15]. Suzuki cross coupling reaction of the precursor DAE and tetra (4-bromobenzoylmethyl) methane I, which was synthesized by four-fold esterification of pentaerythritol with 4-bromobenzoyl chloride (Scheme 2), provided the tetrafunctional DAE cross-linker in its ring-open form (X_ON_) (Scheme 3). Tetra (4-bromobenzoyl-methyl) methane (I), where I refers to the first cross-linker.

To an ice-cooled solution of pentaerythritol (0.23 g, 1.70 mmol, 1 equivalent) and dry triethylamine (1.13 mL, 8.16 mmol, 4.8 equivalent) in 3 mL of dry dichloromethane was added to a freshly prepared solution of 4-bromobenzoyl chloride (1.79 g, 8.16 mmol, and 4.8 equivalent) in 3 mL of dichloromethane dropwise via an addition funnel under an argon atmosphere. The resulting mixture was stirred at room temperature for 21 h. Afterwards, the reaction mixture was diluted with saturated aqueous Na_2_CO_3_ solution. The organic layer was washed with brine, and it was dried over MgSO_4_. The solvent was removed under reduced pressure. The crude mixture was dissolved in dichloromethane and filtrated over a pad of silica. The filtrate was concentrated in vacuum to yield the target compound as a white solid (47%). ^1^H NMR (300 MHz, CDCl_3_): δ 7.84–7.79 (m, 8H, 4×2×C Har), 7.56–7.52 (m, 8H, 4×2×CHar), 4.65 (s, 8H, 4×CH_2_-symm), ^13^C NMR (75 MHz, CDCl_3_): δ 165.4, 132.1, 131.2, 128.9, 128.2, 63.7.

*n*-butyllithium (*n*-BuLi) is widely used as a polymerization initiator in the preparation of elastomers. A solution of *n*-BuLi (1.28 mL, 2.81 mmol, 2.2 M in hexane, 1.1 equivalent) was added dropwise to a solution of the precursor-DAE (747 mg, 2.55 mmol, 1 equivalent) in 4 mL of dry tetra-hydro-furan (THF) in a dry Schlenk flask at room temperature under an argon atmosphere. The reaction mixture turned dark red and was stirred at room temperature for 30 min. Afterwards, tri-isopropyl borate (0.88 mL, 3.83 mmol, 1.5 equivalents) was added and the mixture was stirred for another 1.5 h. Meanwhile, tetra(4-bromobenzoylmethyl)methane I (251 mg, 0.59 mmol, 0.23 equivalent) was dissolved in 4 mL of THF in a 10 mL dry Schlenk flask and tetrakis (triphenylphosphine) palladium(0) (295 mg, 0.26 mmol, 0.1 equivalent) was added in one portion under argon flow. The resulting yellow mixture was stirred at room temperature for 1 h. Then, 5.2 mL of a degassed 2 M aq. Na_2_CO_3_ solution and 1 drop of ethylene glycol were added. The resulting two-phase system was heated to reflux. The resulting borate was added to this solution via a syringe without any work-up. Subsequently, the combined solutions were stirred at 65 °C for 20 h. Afterwards, the reaction mixture was quenched with water, extracted three times with dichloromethane and dried over MgSO_4_. The solvent was removed under reduced pressure. The crude product was purified by column chromatography (petroleum ether: dichloromethane = 1:3) to yield the desired cross-linker X_ON_ as a white solid (36%) ^1^H NMR (500 MHz, toluene-d_8_): δ 8.02 (d, *J* = 8.4 Hz, 8H, 4×2×CHar), 7.31 (d, *J* = 8.4 Hz, 8H, 4×2×CHar), 7.12 (s, 4H, 4×CHthio), 5.74 (s, 4H, 4×CHfur), 4.70 (s, 8H, 4×CH_2__symm), 2.70 (m, 16H, 4×2×CH_2_), 2.05 (s, 12H, 4×CarCH_3_), 1.96 (d, 24H, 2×4×CarCH_3_), 1.95–1.89 (m, 8H, 4×CH_2_); ^13^C NMR (126 MHz, toluene-d_8_): δ 166.0, 150.0, 147.4, 139.7, 139.6, 138.6, 136.4, 133.0, 132.6, 131.2, 129.6, 128.7, 128.6, 126.5, 125.6, 119.0, 107.3, 64.4, 44.0, 39.5, 38.4, 23.6, 14.9, 13.7, 13.6; HRMS (*m*/*z*): [M − H]^−^ calculated for [C_97_H_92_O_12_S_4_], 1575.5393; found 575.6412.

### 2.6. Synthesis of Monomer MIMA and Blank, Linear Polymer P

Atom-transfer radical polymerization (ATRP) (Scheme 2 and Scheme 4) of a furyl-protected maleimide methacrylate (fpMIMA) and lauryl methacrylate (LMA) yields the furan-protectedrandom copolymer poly(LMA–*co*–fpMIMA) fpP, which can be de-protected to the reactive, un-masked poly(LMA–*co*–MIMA) P by heating at 130 °C for 3 h.

The employed masked maleimide methacrylate (fpMIMA) monomer was prepared in three synthetic steps by adapted reported procedures (Scheme 4, Scheme 5 and Scheme 6).

Furan (21.82 mL, 300.0 mmol, 1 equivalent) was added to a solution of maleic anhydride (22.09 g, 225.3 mmol, 0.75 equivalents) in 13 mL ethyl acetate and the reaction mixture was stirred for 24 h at room temperature The obtained white precipitate was filtered off and dried in vacuum to yield mainly the exo-compound as a white solid (65%). ^1^H NMR (300 MHz, DMSO-d_6_): δ 6.59 (t, *J* = 0.9 Hz, 2H, CH=CH), 5.36 (t, *J* = 0.9 Hz, 2H, CH–O–CH), 3.32 (s, 2H, CH–CH); ^13^C NMR (75 MHz, c): δ 171.6, 136.9, 81.7, 49.1, 2-(2-Hydroxyethyl)-3a,4,7,7a-tetrahydro-1H-4,7-epoxyisoindole-1,3(2H)-dione (Scheme 7).

To a suspension of 4, 10-dioxatricyclo [5.2.1.02.6] dec-8-ene-3.5-dione (32.32 g, 194.6 mmol, 1 equivalent) in 58 mL of ethanol, 2-aminoethanol (12.24 mL, 202.4 mmol, 1.04 equivalent) was added dropwise leading to formation of a clear solution. The reaction mixture was heated to 85 °C for 4.5 h and was then allowed to cool to room temperature and stirred for another 12 h. The formed-yield (white precipitate) was filtered off to obtain mainly the exo-compound as a white solid (43%): ^1^H NMR (300 MHz, CDCl_3_): δ 6.51 (t, *J* = 0.9 Hz, 2H, CH=CH), 5.27 (t, *J* = 0.9 Hz, 2H, CH–O–CH), 3.78–3.71 (m, 2H, CH_2_OH), 3.71–3.63 (m, 2H, NCH_2_), 2.88 (s, 2H, CH–CH), 2.42 (br, s, 1H, –OH); ^13^C NMR (75 MHz, CDCl_3_): δ 176.7, 136.4, 80.9, 60.1, 47.4, 41.6, 2-(1,3-Dioxo-3a,4,7,7a-tetrahydro-1H-4,7-epoxyisoindol-2(3H)-yl)ethyl methacrylate (fpMIMA) (Scheme 8).

In a 25 mL Schlenk flask under an argon atmosphere, methacryloyl chloride (0.15 mL, 1.5 mmol, 1.05 equivalent) was added dropwise to a solution of 2-(2-hydroxyethyl) 3a,4,7,7a-tetrahydro-1H-4,7-epoxyisoindole-1,3(2H)-dione (0.31 g, 1.5 mmol, 1 equivalent) and triethylamine (0.25 mL, 1.8 mmol, 1.2 equivalent) in 7 mL of dry dichloromethane at 0 °C. The reaction mixture was stirred for 2 h at 0 °C. The reaction mixture was diluted and extracted with dichloromethane. Then, it was washed two times with an aq. NaHCO_3_ solution and water. After removal of the solvent under reduced pressure, colorless waxy oil was obtained. A short silica column (ethyl acetate:dichloromethane = 4:5) provided a white solid. This solid was identified as the exo-compound of fpMIMA (89%). Then, 4-Methoxyphenol (30 ppm) was added as radical inhibitor before removing the solvent under reduced pressure. ^1^H NMR (300 MHz, CDCl_3_): δ 6.51 (t, *J* = 0.9 Hz, 2H, CH=CH), 6.07 (dd, *J* = 1.6, 1.0 Hz, 1H, C=CH_2_), 5.56 (p, *J* = 1.6 Hz, 1H, C=CH_2_), 5.26 (t, *J* = 0.9 Hz, 2H, CH–O–CH), 4.32–4.24 (m, 2H, OCH_2_), 3.85–3.77 (m, 2H, NCH_2_), 2.86 (s, 2H, O=C–CH–CH–C=O), 1.90 (dd, 3JH, H = 1.6, 1.0 Hz, 3H, CH_3_); ^13^C NMR (75 MHz, CDCl_3_): δ 175.9, 166.9, 136.5, 135.8, 126.0, 80.8, 60.8, 47.4, 37.6 18.1.

The reaction was carried out under inert conditions. Dry toluene was degassed by bubbling argon through the solution for 30 min. Greenish Cu (I) Br was purified several times with acetic acid and subsequently with methanol and then dried in vacuum for at least 12 h. The inhibitor in fpMIMA was removed by filtration over aluminum oxide prior to use. 

Masked maleimide methacrylate (fpMIMA) (0.11 g, 0.40 mmol, 0.16 equivalent) and Cu(I)Br (16 mg, 110 µmol, 0.04 equivalent) were placed in a pressure tube equipped with a magnetic stir bar and kept under vacuum for 1 h. In a dry 25 mL Schlenk flask, lauryl methacrylate (0.74 mL, 2.51 mmol, 1 equivalent), HMTETA (30 µL, 110 µmol, 0.04 equivalent) were dissolved in 2 mL of toluene. Argon was bubbled through the solution for several minutes. Afterwards, the reaction mixture was added to the solids in the pressure tube. After stirring at room temperature for 20 min, the resulting mixture was heated to 70 °C in an oil bath. 

The polymerization was started by adding ethyl α-bromoisobutyrate (EBiB) (16 µL, 110 µmol, 0.04 equivalents) to the solution. The reaction mixture was stirred for 3 h at 70 °C whereas the solution turned greenish. The reaction was stopped subjecting the flask to air and by adding THF (2 mL). The catalyst and ligand were removed by passing through a basic aluminum oxide column, followed by a removal of the solvent under reduced pressure. The residue was dissolved in a minimum amount of toluene and precipitated in ice-cold methanol several times. This was done to afford poly(LMA–*co*–fpMIMA) (fpP) (Scheme 9) as a colorless viscous oil ^1^H NMR (300 MHz, CDCl_3_): δ 6.54 (s, br, –CH=CH–, furyl moiety), 5.28 (s, br, CH–O–CH), 3.90 (s, br, O–CH_2_, LMA side chain), 3.75 (s, br, O–CH_2_, N–CH_2_, MIMA), 2.98 (s, br, O=C–CH–CH–C=O), 1.89 (s, br, CH, polymer backbone, MIMA), 1.79 (s, br, CH, polymer backbone, LMA), 1.61 (s, br, O–CH_2_–CH_2_–, LMA side chain), 1.27 (s, br, (CH_2_)_9_, LMA side chain), 1.12 (s, br, CH_3_, polymer backbone, MIMA), 1.02 (s, br, CH_3_, polymer backbone, LMA), 0.90–0.86 (t, br, CH_3_, LMA side chain); ^13^C NMR (126 MHz, CDCl_3_): δ 179.7, 177.6, 176.8, 138.1, 80.6, 64.8, 61.4, 54.0, 47.3, 44.8, 37.7, 31.7, 29.4, 29.3, 29.1, 27.9, 25.8, 22.4, 14.0: SEC (THF, 40 °C) of the prepared polymers gave a number average molecular weight n between 6000 and 8600 g·mol^−1^ and a dispersity Đ between 1.17 and 1.26. The amount of masked maleimide methacrylate fpMIMA was determined via integration and comparison of diagnostic peaks in the NMR spectra and amounts to 2 × 10^−1^ mol %.

Poly(LMA–*co*–MIMA) (P) (Scheme 10).

A bulk film of poly (LMA–*co*–fpMIMA) fpP was heated on a glass substrate in a drying oven at 130 °C for 3 h. ^1^H NMR analysis showed quantitative conversion of the oxabicyclic moiety to the maleimide functional group to obtain de-masked poly(LMA–*co*–MIMA) P. ^1^H NMR (300 MHz, CDCl_3_): 6.80 (s, br, CH=CH, MIMA side-chain), 3.91 (s, br, O–CH_2_, LMA side-chain), 3.82 (s, br, O–CH_2_, N–CH_2_, MIMA), 1.91 (s, br, CH, polymer backbone, MIMA), 1.80 (s, br, CH, polymer backbone, LMA), 1.61 (s, br, O–CH_2_–CH_2_–, LMA side-chain), 1.27 (s, br, (CH_2_)_9_, LMA side-chain), 1.13 (s, br, CH_3_, polymer backbone, MIMA), 1.03 (s, br, CH_3_, polymer backbone, LMA), 0.90–0.86 (t, br, CH_3_, LMA side-chain); ^13^C NMR (75 MHz, CDCl_3_): δ 178.1, 177.4, 170.3, 134.3, 65.0, 61.4, 48.1, 43.4, 38.8, 32.2, 29.9, 29.8, 29.6, 28.4, 26.2, 23.0, 14.3.

Besides NMR measurements, the de-protection from fpP to P was monitored via FT-IR spectroscopy as well as thermogravimetric analysis (TGA) and differential scanning calorimetry (DSC).

## 3. Results

### 3.1. Preparation of Linear Polymer and Cross-Linker

More than one reactive furyl moiety can carry out an efficient cross-linking processes when using chains of linearly connected polymer hence we can use a tetra-functional motif X. Thus, one reduces the necessary and sufficient quantity of cross-linkers to complete the reaction. This allows achieving the upper limit of maximum light penetration [21]. In addition, the mechanism of attracting electrons at the contact-surface of the diarylethene to the pentaerythritol bulk could get ester groups with high photo-chemical efficiency and elevated fatigue resistance [22]. Here, one can keep the advantages of a possibility to activate the dynamic bond on demand and to increase the capacity to switch “off” the unreacted cross-linker. In Figure 1, one can see the right side of the scratched-sample irradiated during 30 min with a LED-365 nm (under argon ambient) has changed (Figure 1a–c) through the UV-irradiation (Figure 1b). Then, we notice the complete disappearance of the scratch in Figure 1e. One can notice in Figure 1b,c (right side) that local irradiation (using UV) forms a static polymer network that repressed the scratched-singes on the sample.

### 3.2. Mechanical Properties of Linear Polymer P and Polymer Networks

For the mechanical properties, we present the shear storage │*G’*│ and shear loss │*G”*│ as a function of temperature, *T*, of X#P_ON_ (dynamic) and X#P_OFF_ (static) in Figure 2a, while Figure 2b shows the viscosity coefficient, η, as a function of *T*.

Temperature-dependence of the complex viscosity │η│* of blank sample P (gray line Figure 2a) and polymer networks X#P_ON_ (blue → green line, Figure 2a) and X#P_OFF_ (yellow line, Figure 2a) (heating at 0.02 K·s^−1^) are valid in a temperature range of 40 to 105 °C: │η│* (X#P_ON_) ≈ │η│* (X#P_OFF_) │η│* (P). The polymer networks X#P_ON_ and X#P_OFF_ in that low temperature range reveal a drastically increased complex viscosity in contrast to the blank, linear polymer P valid in a temperature range of 117 to 130 °C. One can write:

│η│*·(P) ≈ │η│*·(X_ON_ + P) ≈ {2│η│*·(X#P_OFF_)}

Only the complex viscosity of X#P_ON_ reaches the mean values of P upon heating to temperatures higher than ca. 110 °C. In strong contrast, the complex viscosity of locked network X#P_OFF_ remains higher than X#P_ON_ and P, thus different material properties occur in a high temperature region confirming the light-induced locking and de-locking of the material’s cross-link density.

### 3.3. Temperature-Controlled Sol–Gel Transition in X#P_ON_

As seen in Figure 3, we applied a constant normal force of 0.2 N for gap control. Heating ramps were conducted at ca. 0.5 K·s^−1^ utilizing a Peltier element and collecting data points every 7 to 15 s with three repetitions per data point. Data analysis was performed with the software HAAKE RheoWin 4.3 (HAAKE™ Thermo Electron, Newington, NH, USA). Rheological data were smoothed using the Adjacent-Averaging Method (OLCN-USA), except for graphs in Figure 3. Note that compression or tensile measurements could not be performed due to the film’s high viscoelasticity and creep even at low temperature. The procedure for polymer network preparation of X#P_ON_ was equal to typical scratching tests, followed by pestling the bulk material in liquid nitrogen media and storing for 16 h under low pressure atmosphere to obtain a powder of X#P_ON_. Recording FT-IR spectra before and after milling shows no changes, proving no structural destruction of the material. The ^1^H MAS spectrum shows two strong signals at δ = 0.88 ppm and δ = 1.28 ppm belonging to the predominating protons of the poly(lauryl methacrylate) backbone (see Figure 3b). However, due to overlapping and rather broad signals, a quantification to determine the amount of cross-linking efficiency could not be carried out.

### 3.4. FT-IR Spectroscopic Analysis of the De-Protection of Furyl-Protected, Inactive Linear Polymer fpP to Form Non-Protected, Active Linear Polymer P via Cleavage of the Furan Protection Group

The network formation has been studied from a kinetic point of view. The illumination time during cross-linking of furan modified with maleimide was studied as a function of the amount of furan. Figure 4a illustrates complete FT-IR spectra of fpP and of P before (black solid line and after heating of fpP in the bulk to 130 °C in a drying oven for 1 h, gray dashed line). Spectra are normalized with respect to the band at 2923 cm^−1^. In Figure 4b, we zoomed in on the C=O stretching mode of the succinimide moiety in the Diels–Alder adduct [2,3,23] in fpP at 1778 cm^−1^ as well as c, the out of plane CH-bending mode of the vinylene group of the furyl moiety [14,24] at 855 cm^−1^.

### 3.5. Differential Scanning Calorimetry Measurements of Polymer Networks X#P_ON_ and X#P_OFF_

In differential scanning calorimetry measurements, the de-cross-linking of the unlocked polymer network X#P_ON_ and the locked network X#P_OFF_ was recorded as an endothermic peak due to the removal of cross-linking points caused by the endothermic retro Diels–Alder reaction in a temperature range of 90 to 180 °C (Figure 5). The energy required for the endothermic de-cross-linking reaction, i.e., the reaction enthalpy ∆*HR*, can be quantified by integrating the area of the respective peak 2, 25. In X#P_OFF_, a number of cross-linking points are being locked by UV-light and hence the retro Diels–Alder reaction is inhibited at these sites. The respective endotherm is, therefore, lowered and the associated smaller integral of the corresponding peak in the DSC curves confirms the reduced reaction enthalpy. Assuming a more or less homogeneous distribution of cross-linking points, the relative amount of cross-linking points, which are locked upon UV-light illumination, can be estimated by the ratio of the measured reaction enthalpies. In the first heating cycle, the integrated area in X#P_OFF_ is 33% lower (peak area = 82.9 mJ, ∆*HR* = 9.3 J·g^−1^) than in X#P_ON_ (peak area = 123.8 mJ, ∆*HR* = 13.6 J·g^−1^) (Figure 5). In the second heating cycle, a difference of 38% is calculated (for X#P_ON_: peak area = 82.3 mJ, ∆*HR* = 9.0 J·g^−1^; for X#P_OFF_: peak area = 51.3 mJ, ∆*HR* = 5.7 J·g^−1^) confirming the result of the first heating cycle. Thus, it can be assumed, that around 1/3 of the cross-linking points are locked and cannot undergo the de-cross-linking reaction in the bulk material. 

Figure 5 shows DSC measurements of fpP 55, including (Figure 5a) a strong endothermic peak at 120 to 180 °C (retro Diels–Alder reaction and evaporation of furan) and (Figure 5b, inset) in the first heating curve. In the second heating curve, another endothermic peak cannot be observed.

Figure 5b displays the thermogravimetric analysis (TGA) of fpP showing a mass loss of the furan protection group in b’. 

### 3.6. UV Irradiation of Polymer Chains

Figure 6 shows the UV/visible absorbance of polymer chain where there is almost no change before and after absorbance. One can get more reactive groups (under desire) by using variable amounts of maleimide and we can adjust the process to get the maximum cross-linking density. This is achieved by using linear chains of maleimide functionalized poly (lauryl methacrylates) in such a way that P (*Mn* = 6000–8600 g·mol^−1^). Synthesis of reactive-groups occurs by atom transfer radical polymerization with narrow dispersity (Ð = 1.17 − 1.26). 

This is due to the introduction of dodecyl part chains in the polymer fundamental-corner and therefore some reflows and rearrangements occur through the material-matrix. 

### 3.7. Scratching Tests of X#P (without Light Control) Upon Variation of Cross-Linking Density

When we illuminate only a small portion of the scratched sample using UV, we will notice the creation of a static polymer network due to the thermos reversibility of this dynamic system. Similarly, instead of illumination with UV, we use visible light. Figure 1c,d illustrates the ease of healing by illumination with visible light. In a successive manner, we repeated this process for different cycles, which shows a complete reversibility of all involved steps. Figure 7 shows some scratching tests including blank sample P without cross-linker. 

#### Scratching Tests of the Bulk Material of Blank Sample P without Cross-Linker

For this purpose, a bulk film of poly(LMA–*co*–fpMIMA) (fpP) was heated at 130 °C for 3 h to cleave the furan protection group to form poly(LMA–*co*–MIMA) (P), followed by tempering at 40 °C for additional 16 h. Afterwards, a model scratch was done with a scalpel in a controlled manner in the mm scale. 

Disappearance of the scratch at room temperature was followed by optical microscopy at different time intervals. For preparation of a film of X#P_ON_, furyl-protected copolymer (fpP) and cross-linker X were dissolved in a minimum amount of dichloromethane and drop-casted onto a glass slide. The mixture was heated at 130 °C for 3 h, followed by annealing at 40 °C for 16 h. Then, the surface of the polymer network X#P_ON_ was scratched in a controlled manner. Healing of the scratch at different temperatures was followed by optical microscopy. 

### 3.8. Determination of the Conversion of the Diels–Alder Cross-Linking Reaction of X#P_OFF_ in the Photo Stationary State via UV/Visible Spectroscopic Analysis

Domination of the healing capacity within scratched samples of X#P_ON_ is a simple technique to study local control over the thermal healing process. In order to get minimum values of the optical density, we take 11 mol % maleimide content containing four furyl groups and P. Then, we mixed them in quantities to get 0.7 equivalents of furyl groups per maleimide unit, which minimizes the optical density. Moreover, Figure 8 shows that the cross-linking technique transfer about 87% of the furyl groups by ultraviolet/visible spectroscopy. In addition, Figure 9 confirms these results using solid state ^1^H NMR experimental data.

### 3.9. UV-Vis Spectroscopy of Unlocked Polymer Network X#P_ON_

In order to perform solid state UV/vis-spectroscopy of blank sample (P) measurements, we span 3–5 µL of a solution of free cross-linker X_ON_ and the respective polymer in degassed (THF) on 1 × 1 cm^2^ quartz glass plates. We used AFM measurements in tapping mode to measure the thickness: thickness of plates is 1 mm and thickness of polymer film is approximately 2.0 µm

One notes that there is no cross-linker for blank sample preparation and there are 0.6 and 0.7 equivalent furan per maleimide unit. Spin coating was performed at a rotation speed of 100–150 rps with a spin coating time set to 60 s with a KLM spin coater SCC-200 from SCHAEFER Technologies Corporation (Langen, Germany) at room temperature. Thermal cross-linking was carried out for 16 h at room temperature. Irradiation was performed directly in a Varian Cary 50 UV/visible spectrophotometer (Agilent, Santa clara, CA, USA) equipped with a Peltier thermos-stated cell holder at 25 ± 0.05 °C by adjusting the LED in a distance of 1 cm orthogonal to the quartz glass plate in the sample holder. A Roithner 365 nm-LED XSL-365-5E for ring-closing at 20 mA and 4.2 V and a LED Engin 460 nm-Blue LED Emitter LZ4-00B208 (Roithner Laser TecchnikGmbH, Vienna, Austria) for ring-opening at 2–3 mA and 12 V were employed, both driven by a GW Instek GPD-3303S linear DC power (Taipei, Taiwan) supply.

### 3.10. UV/Visible Spectra for Determination of the Photo-Conversion of X#P_OFF_ in the Photo-Stationary State

Photo-conversion of X#P_OFF_ in the photo-stationary state UV/visible spectra of a small molecule reference compound, either in its 100% ring-open or in its 100% ring-closed state (Ref_OFF_, yellow dashed line) were recorded in degassed acetonitrile (*c* ≈ 10^−5^ M). The UV/visible spectrum of X#P_ON_ (blue solid line) is normalized to the peak maximum of Ref_ON_ at 330 nm (where the blank sample P absorbs insignificantly). The thus derived factor is used to normalize X#P_OFF_, so that the maxima of the diagnostic bands of X#P_OFF_ and Ref_OFF_ can be compared with respect to the amount of formed ring-closed Diels–Alder adduct. This analysis indicates ca. 83% photo-conversion of X#P_OFF_ in the photo-stationary state in thin films (Figure 10). Note that this value represents an upper limit of the amount of ring-closed isomer in the PSS and it should be lower in thicker films due to reduced optical penetration. Polymer film thickness for UV/visible spectroscopical measurements is approximately 2.0 µm, determined by AFM measurements in the tapping mode.

### 3.11. Small-Angle X-ray Scattering Curves of the Copolymer P without Cross-Linker X_ON_

A curve fit for interpretation of the scattering curve of X#P_ON_ using *I* (q) is given exemplarily (blue dashed line, see Equation (2) and [25]). The cyan dashed line represents the scattering contribution *I*_1_ (*q*) from large inhomogeneities with sizes ≥52 nm, the green solid curve is the scattering contribution *I*_2_ (*q*) from the polymeric mesh, and the magenta dash-dotted curve represents the scattering contribution *I*_3_ (*q*) from the broad peak. Polymer networks produce characteristic SAXS (small-angle X-ray scattering) patterns, which provide information on their structure according to the theory originally derived by de Gennes [26] and further developed by Panyukov and Rabin [27]. 

Hence, we assume that the scattering pattern differs among the different states of the polymeric network structure. Accordingly, changes of the polymeric mesh in network X#P_ON_, X#P_OFF_ and reestablished X#P_ON_ at room temperature as well as after heating to the retro Diels–Alder reaction temperature were determined via small angle X-ray scattering. 

## 4. Discussion

We assume that the scattering pattern differs among the different states of the polymeric network structure. Accordingly, changes of the polymeric mesh in network X#P_ON_, X#P_OFF_ and reestablished X#P_ON_ at room temperature as well as after heating to the retro Diels–Alder reaction temperature were determined via small angle X-ray scattering. Resultant scattering curves and appropriate mesh sizes are compared in Figure 11 and see Table 1, Table 2, Table 3, Table 4 and Table 5. First, the resultant scattering curves of blank linear polymer P without added cross-linker (gray solid line, Figure 11) and the curve of unlocked cross-linked polymer X#P_ON_ (black solid line) are compared at 21 °C to clarify all scattering contributions as well as the difference between non-cross-linked and cross-linked material at ambient temperature. We assign three characteristic regions in the scattering pattern of cross-linked X#P_ON_, labeled as 1, 2 and 3 (Figure 11), whereas in the scattering curve of linear polymer P only scattering contributions 1 and 3 occur. 

### 4.1. Scattering Contribution 1

Region 1 is dominated by a forward scattering, *I*_1_ (*q*), with a sharp increase at *q*-values lower than 0.2 nm^−1^. The cyan dashed line (Figure 10) represents the curve fit of scattering contribution *I*_1_ (*q*) in X#PON. *I*_1_ (*q*) can be interpreted as resultant from large scale inhomogeneities of the bulk polymers and is present in cross-linked X#P_ON_ and linear P. Tentatively, it should be characterized by a first correlation length δ_1_.

### 4.2. Scattering Contribution 2

The second scattering contribution, *I*_2_ (*q*), can be interpreted as resultant from the network and is characterized by its entanglement distance. The contribution of *I*_2_ (*q*) is clearly visible in the total scattering of the cross-linked polymer X#P_ON_ between 0.3 nm −1 < *q* < 1.2 nm^−1^. The green solid line (Figure 11) represents the curve fit of scattering contribution *I*_2_ (*q*) in X#P_ON_ which is approximately three times larger than the scattering of non-cross-linked P. We interpret this as a characteristic of the network X#P_ON_, which is not present in linear P. Therefore, the mesh size of this network can be described by a second correlation length δ_2_.

### 4.3. Scattering Contribution 3

Region 3 of the scattering pattern is dominated by a broad peak, *I*_3_ (*q*), with a maximum at *q*_max_ around 2.5 nm^−1^ and is fitted by a magenta dash-dotted curve (Figure 10). This broad peak is present in the scattering pattern of X#P_ON_ as well as in P and is therefore not a characteristic of the network. The presence of such a peak is well known for concentrated polymer systems that display micro-phase separation such as block copolymers in the amorphous state [28,29]. The underlying physical effect is referred to as “correlation-hole” effect. A reasonable interpretation for the presence of the same peak in network X#P_ON_ as well as in linear P is to assume that the dodecyl chains of the poly(lauryl methacrylate) backbone are micro-phase separated from the polymer backbone in these domains. The maximum diameter of these alkyl chain rich domains can be estimated [30] as two-times the alkyl chain lengths, which is 2*l*_c_ = (11 × 0.1265 + 0.15) nm = 3.08 nm. We quantified the broad peak by a characteristic distance of *d* = 2π/*q*_max_ and a correlation length δ_3_.

### 4.4. Physical Background and Discussion of Results for X#P_ON_ and P

Taking all effects into account, we approximate the total scattering *I* (*q*) as a sum of the three scattering contributions.

(1) $$I(q)=I_{1}(q)+I_{2}(q)+I_{3}(q)$$

In particular, the Debye–Büche function is used for *I*_1_ (*q*), the Ornstein-Zernike function for the cross-linking contribution *I*_2_ (*q*) and a Lorentzian peak function for *I*_3_ (*q*), resulting in:

(2) $$I(q)=\frac{k_{1}}{{\left[1+{\left(\xi_{1}q\right)}^{2}\right]}^{2}}+\frac{k_{2}}{{\left[1+{\left(\xi_{2}q\right)}^{2}\right]}^{2}}+\frac{k_{3}}{{\left[1+{\left(\xi_{3}|q-q_{\max}|\right)}^{2}\right]}^{2}}$$

with scaling parameters *k*_1_, *k*_2_, and *k*_3_ representing the maximum contribution to the respective scattering intensity correlation lengths *δ*_1_, *δ*_2_, and *δ*_3_; and *q*_max_ as the peak position. Matsunaga et al. [31] have applied the approach of utilizing the first two terms for the interpretation of small-angle neutron scattering data of tetra-arm PEG gels. We refer to their study and references therein [32] for a more detailed discussion of the scattering of polymeric gels as the most studied polymeric networks. During the fitting procedure, we found ambiguous values for δ_1_ because it is larger than our limit of determination. The maximum size available is given as = π/*q*_min_. From the smallest *q*-value of *q*_min_ = 0.06 nm^−1^ we determined = π/*q*_min_ of 52 nm. This value was used as fixed parameter for all curve fittings to avoid ambiguous results. It should be noted that polymer networks often exhibit a hierarchical structure, with the largest dimensions on a length scale of greater than 100 nm, which is not accessible with SAXS. Here, USAXS (ultra small-angle X-ray scattering) is a useful technique that allows obtaining information on structure hierarchy, as described by Zhang and Ilavski [33]. However, USAXS was not used in the present study and information on structure hierarchy is not available. Nevertheless, we found good fit results using *I* (*q*) with the remaining parameters for the cross-linked polymer X#P_ON_ at 21 °C as shown in Figure 10. The second correlation length of X#P_ON_, i.e., the correlation length of the mesh of X#P_ON_, has a mean value of δ_2_ = (1.21 ± 0.07) nm. The parameter values of the peak are δ_2_ = (0.76 ± 0.03) nm and *q*_max_ = (2.69 ± 0.02) nm^−1^, which corresponds to a distance of *d* = 2.33 nm at 21 °C. 

### 4.5. X#P_ON_ at Room Temperature and at 120 °C

Comparison of the scattering curves of X#P_ON_ at 21 °C and after 30 min at 120 °C reveals a shift of scattering contribution 2 to lower *q*-values, and thus, an increase of the correlation length from δ_2_ = (1.21 ± 0.07) nm at 21 °C to δ_2_ = (1.97 ± 0.20) nm at 120 °C. We interpret this finding as a widening of the mesh size by δ_2_ = (0.76 ± 0.21) nm and conclude that at 120 °C the occurrence of a retro Diels–Alder reaction strongly reduces the number of cross-links (X#P_ON_ → X_ON_ + P) (see Table 2). This is supported by the results of the scattering curves of cross-linked X#P_ON_ and linear P where scattering contribution 2 is not present in non-cross-linked P. The broad peak also shifts to a higher value of *q*_max_ = (2.95 ± 0.02) nm^−1^, which corresponds to *d* = 2.13 nm, and broadens which reflects in a lower correlation length of δ_3_ = (0.65 ± 0.02) nm. This finding seems to be a contradiction at first sight. The UV-light induced ring closure shortens the molecular length of the diarylethene units and should therefore intuitively also reduce the correlation length δ_2_. Nevertheless, we tentatively assume that ring-closure has a higher probability at small meshes of the network due to a higher cross-linking and hence a higher photo-switch concentration (see Table 1). For this reason, the mean mesh size can increase due to an apparent disappearance of smaller meshes, as they fall below the SAXS lower size detection limit of *d*_min_ = *p*/*q*_max_ > 0.7–0.8 nm. The scattering intensity becomes too noisy at scattering vectors larger than −1. Furthermore, with SAXS, it is not possible to distinguish between a mesh resulting from chemically cross-linked polymer chains or from physical entanglements of chains or a mixture of both. Thus, we must assume that a physical reorganization of the network structure is also included (for a detailed investigation of this nano structural complexity, see [34].

## 5. Conclusions

Micro damages and cracks lead to structural failure and the ability to heal these defects enables polymers to have high efficiency, less maintenance and longer lifetimes. Polymeric structural materials with hidden damage and micro cracking are not suitable for recent high technology applications. One can easily overcome this problem and repair these defects by self-healing techniques. The experimental data in the present study show that certain photon energy that are coming from light (or UV) affect directly the samples and result in energy-light stimulated and controlled locking (OFF) and de-locking (ON) cycle in complete coincidence with X#P_ON_ as created via simple transformation. Therefore, the present study developed a suitable technology with structural polymeric material, which has the ability to self-heal cracks (and damages) and recover structural function. In particular, this technology could have a substantial advantage in thermosetting-polymers. These polymers have great range of different applications such as aerospace, bio-medical technology, micro-electronics, etc. In addition, the present ideas are valid for a wide variety of brittle compounds such as glasses, chalcogenides, ceramics, etc. In fact, the domain of self-healing is a promising area that can lead to biomimetic healing and one could transport the necessary building blocks and chemicals of healing to the exact location of crack. The proposed technique permits one to transform certain areas strongly and reversibly from a thermally healable dynamic to a static “locked” polymer network. This can be achieved in forward or reversed manner by locally applying light having various wavelengths. Our experimental data confirm that the presented conditional healing really has its origin in the generation and self-cut (scission) of covalent bonds using retro-Diels–Alder reaction. Interestingly, the material was kept safe during this photo-switchable locking and unlocking due to stopping continuous irradiation. In fact, because of an enhanced material mobility necessary for repair, the combination of light stimulation with subsequent thermal healing leads to better healability. We suggest that our reactant system would be adapted to different types of more complex, responsive polymer systems. In addition, the accompanied external control over local dynamic cross-linking has to help the design of repairable soft and biomaterials for a multitude of future applications; for example, healable paints (macroscopic application), and as inherent resistances, which can be carried via different processing steps until being activated to offer control over nanofabrication (microscopic application).

## Figures and Tables

**Scheme 1:** Synthesis of cross-linker X_ON_ (tetrafuryl-substituted DAE-type cross-linker X_ON_).

**Scheme 2:** Four-fold esterification of pentaerythritol with 4-bromobenzoyl chloride.

**Scheme 3:** Tetrafunctional photo-switchable cross-linker in reactive ring-open form (X_ON_).

**Scheme 4:** Synthesis of monomer MIMA.

**Scheme 5:** Synthesis of monomer MIMA.

**Scheme 6:** Synthesis of monomer MIMA, 3a,4,7,7a-tetrahydro-4,7-epoxyisobenzofuran-1,3-dione.

**Scheme 7:** Synthesis of monomer MIMA.

**Scheme 8:** Synthesis of monomer MIMA.

**Scheme 9:** Synthesis of monomer MIMA.

**Scheme 10:** Synthesis of monomer MIMA.

**Figure 1:** ((**a**,**b**) static system) The RS of the scratched-sample irradiated during 30 min. ((**b**,**c**) static system-(X#P_OFF_) One fixed the scratch on heating for 5 min. ((**c**,**d**) static/dynamic system) Healing ability on the left side (X#P_ON_) is kept switched “on” and after irradiation, for 1.5 h. ((**d**,**e**) dynamic system) Micrographs of a scratched dynamic after heating for 5 min. ((**a**,**e**) dynamic system) Illustration of micrographs of a scratched dynamic cross linker (X#P_ON_ thin film) with and without light control.

**Figure 2:** (**a**) Shear storage │G’│ and shear loss │G”│as a function of temperature of X#P_ON_ (dynamic) and X#P_OFF_ (static); and (**b**) viscosity coefficient, η, of locked cross-linker (orange curve) as a function of *T*.

**Figure 3:** Temperature-controlled sol–gel transition in X#P_ON_: Rheological monitoring the thermally reversible re-cross-linking of X_ON_ + P → X#P_ON_; i.e., the Diels–Alder reaction, at constant temperatures (25, 40 and 60 °C) over time. Note that previous de-cross-linking until an equilibrium of G’ and G” with was performed at 124 °C for 30 min. Heating rate to reach constant re-cross-linking temperature: Approximately 0.5 K s^−1^. (**a**) Evolution of G’ and G” during re-cross-linking at 25 °C. The crossover point, where, is reached after *t*_x_ = 670 min and can be attributed to a changing of the viscoelastic properties from a liquid to a solid, i.e., a recovery of the network properties beyond the crossover point. Noteworthy, both moduli already increase strongly within the first few minutes, due to the fast beginning of the network formation. (**b**) At 40 °C the crossover point is already reached after 213 min and (**c**) at 60 °C after 19 min the correlation between temperature *T* and crossover time *t*_x_ is represented in (**d**) confirming the dynamics of the Diels–Alder and retro Diels–Alder reaction, i.e., cross-linking and de-cross-linking. Note that rheology measurements depicted in (**a**–**c**) furthermore confirm a thermos reversibility of the polymeric network due to a usage of the same sample. Full recovery of cross-linking points at 25 and 40 °C can be observed.

**Figure 4:** (**a**) Complete FT-IR spectra of fpP (before heating, black solid line) and of P (after heating of fpP in the bulk to 130 °C in a drying oven for 1 h, gray dashed line). Spectra are normalized with respect to the band at 2923 cm^−1^. (**b**) Zoom in of the C=O stretching mode of the succinimide moiety in the Diels–Alder adduct [2,3,23] in fpP at 1778 cm^−1^ as well as (**c**), the out of plane CH-bending mode of the vinylene group of the furyl moiety at 855 cm^−1^, both not visible in P. For further characterization of P see Figure 1.

**Figure 5:** (**a**) Differential scanning calorimetry (DSC) of fpP; and (**b**) thermogravimetric analysis (TGA) P and b.

**Figure 6:** Dashed line represents UV- or visible-spectra before irradiation and solid line represents the spectra of P after irradiation.

**Figure 7:** (**a**) Photographs showing the disappearance of a model scratch at room temperature after 10 min; and (**b**) the mending of a model scratch after exposing the scratched material to light. (**c**) Low cross-linking density: Photographs showing the mending of a model scratch in X#P_ON_ at 60 °C. (**d**) Higher cross-linking density: Photographs showing non-healable scratches in X#P_ON_ at 120 and 160 °C.

**Figure 8:** UV/visible spectra of X#P_OFF_, partially (magenta line) and the respective Gaussian fits of X_OFF_ (red line with filled area) and X#P_OFF_ (yellow line with filled area).

**Figure 9:** Solid-state ^1^H NMR spectroscopy of unlocked, non-illuminated polymer network X#P_ON_: (**a**–**c**) ^1^H MAS NMR spectrum with two zoom in spectra of X#P_ON_. (**a**) Complete 1H MAS NMR spectrum of X#P_ON_. (**b**) Zoom-in highlighting the peaks related to the poly (lauryl methacrylate) backbone. (**c**) Further zoom-in to peaks belonging to protons of Diels–Alder adduct type cross-linking motifs.

**Figure 10:** UV/visible spectra of X#P and X#P (solid lines) in comparison to a small molecule reference compound (dashed lines) in its 100% ring-open state (Ref_OFF_) and 100% ring-closed state (Ref_ON_).

**Figure 11:** Small-angle X-ray scattering patterns for different scatterings. Scattering curves of the copolymer P without cross-linker X_ON_ (gray solid line) and as part of polymer network X#P_ON_ (black solid line) measured at 21 °C.

**Table 1:** Overview over mesh sizes of unlocked polymer network X#P_ON_ at 21 °C and of locked polymer network X#P_OFF_ formed after UV-light illumination described by a second correlation length δ_2_ with added explanation. Mesh sizes are determined by SAXS measurements.

Correlation Length	X#P_ON_ at 21 °C	X#P_OFF_ at 21 °C	∆ δ_2_ (nm)
**δ_2_ (nm)**	**1.21 ± 0.07**	**1.61 ± 0.10**	**→ 0.40 + 0.10**

Higher probability of ring-closure at small mesh sizes which disappear → widening of mesh size.

**Table 2:** Overview over mesh sizes of unlocked polymer network X#P_ON_ at 120 °C for 30 min to form X_ON_ + P described by a second correlation length δ_2_ with added explanation. Mesh sizes are determined by SAXS measurements.

Correlation Length	X#P_ON_ at 21 °C	X#P_OFF_ at 21 °C	∆ δ_2_ (nm)
**δ_2_ (nm)**	**1.21 ± 0.07**	**1.97 ± 0.20**	**→ 0.67 + 0.21**

Reduction of number of cross-links upon heating **→** widening of mesh size.

**Table 3:** Overview over mesh sizes of locked polymer network X#P_OFF_ at 21 °C and at 120 °C for 30 min described by a second correlation length δ_2_ with added explanation. Mesh sizes are determined by SAXS measurements.

Correlation Length	X#P_OFF_ at 21°C	X#P_OFF_ at 120 °C	∆ δ (nm)
**δ_2_ (nm)**	**1.61 ± 0.10**	**1.91 ± 0.10**	**→ 0.30 + 0.10**

Successful locking of cross-linking points upon heating → only slight.

**Table 4:** Overview over mesh sizes of locked polymer network X#P_OFF_ at 21 °C and of reestablished unlocked polymer network X#P_ON_ reformed after visible-light illumination described by a second correlation length δ_2_ with added. Mesh sizes are determined by SAXS measurements.

Correlation Length	X#P_OFF_ at 21°C	X#P_OFF_ at 120 °C	∆ δ_2_ (nm)
**δ_2_ (nm)**	**1.61 ± 0.10**	**1.91 ± 0.10**	**→ 0.30 + 0.10**

Higher probability of ring-opening at small mesh sizes upon visible-light illumination with appearance of smaller meshes in mean mesh size → decrease of mesh size → successful restoration of mesh sizes of original; X#P_ON_ → only slight.

**Table 5:** Overview over mesh sizes of reestablished unlocked polymer network X#P_ON_ at 21 °C and after heating to 120 °C for 30 min to form X_ON_ + P described by a second correlation length δ_2_ with added explanation. Mesh sizes are determined by SAXS measurements.

Correlation Length	X#P_OFF_ at 21°C	X#P_OFF_ at 120 °C	∆ δ_2_ (nm)
**δ_2_ (nm)**	**1.27 ± 0.11**	**1.93 ± 0.12**	**→ 0.66 + 0.12**

Reduction of number of cross-links upon heating → widening of mesh size.
